The article "Longitudinal Data From the KETO-CTA Study: Plaque Predicts Plaque, ApoB Does Not" was retracted in 2026. Reasons: unreliable data; concerns about the methods.

# Longitudinal Data From the KETO-CTA Study: Plaque Predicts Plaque, ApoB Does Not

**DOI:** 10.1016/j.jacadv.2025.101686

**Published:** 2025-04-07

**Authors:** Adrian Soto-Mota, Nicholas G. Norwitz, Venkat S. Manubolu, April Kinninger, Thomas R. Wood, James Earls, David Feldman, Matthew Budoff

**Affiliations:** a Metabolic Diseases Research Unit, National Institute for Medical Sciences and Nutrition Salvador Zubiran, Mexico City, Mexico; b Tecnologico de Monterrey, School of Medicine, Mexico City, Mexico; c Harvard Medical School Boston, Massachusetts, USA; d Lundquist Institute at Harbor-UCLA Medical Center, Torrance, California, USA; e Department of Pediatrics, University of Washington School of Medicine, Washington, USA; f Cleerly, New York, New York, USA; g Citizen Science Foundation, Las Vegas, Nevada, USA

**Keywords:** ApoB, atherosclerosis, body mass index, coronary computed tomography angiography, carbohydrate-restricted diet, ketogenic diet, LDL cholesterol, lean mass hyper-responder, saturated fat

## Abstract

**Background:**

Changes in low-density lipoprotein cholesterol (LDL-C) among people following a ketogenic diet (KD) are heterogeneous. Prior work has identified an inverse association between body mass index and change in LDL-C. However, the cardiovascular disease risk implications of these lipid changes remain unknown.

**Objectives:**

The aim of the study was to examine the association between plaque progression and its predicting factors.

**Methods:**

A total of 100 individuals exhibiting KD-induced LDL-C ≥190 mg/dL, high-density lipoprotein cholesterol ≥60 mg/dL, and triglycerides ≤80 mg/dL were followed for 1 year using coronary artery calcium and coronary computed tomography angiography. Plaque progression predictors were assessed with linear regression and Bayes factors. Diet adherence and baseline cardiovascular disease risk sensitivity analyses were performed.

**Results:**

High apolipoprotein B (ApoB) (median 178 mg/dL, Q1-Q3: 149-214 mg/dL) and LDL-C (median 237 mg/dL, Q1-Q3: 202-308 mg/dL) with low total plaque score (TPS) (median 0, Q1-Q3: 0-2.25) were observed at baseline. The median change in NCPV was 18.9 mm^3^ (IQR: 9.3-47.0 mm^3^) and the median change in PAV was 0.8% (IQR: 0.3%-1.7%). Neither change in ApoB (median 3 mg/dL, Q1-Q3: −17 to 35 mg/dL), baseline ApoB, nor total LDL-C exposure (median 1,302 days, Q1-Q3: 984-1,754 days) were associated with the change in noncalcified plaque volume (NCPV) or TPS. Bayesian inference calculations were between 6 and 10 times more supportive of the null hypothesis (no association between ApoB and plaque progression) than of the alternative hypothesis. All baseline plaque metrics (coronary artery calcium, NCPV, total plaque score, and percent atheroma volume) were strongly associated with the change in NCPV.

**Conclusions:**

In lean metabolically healthy people on KD, neither total exposure nor changes in baseline levels of ApoB and LDL-C were associated with changes in plaque. Conversely, baseline plaque was associated with plaque progression, supporting the notion that, in this population, plaque predicts plaque but ApoB does not. (Diet-induced Elevations in LDL-C and Progression of Atherosclerosis [Keto-CTA]; NCT05733325)

Carbohydrate-restricted diets (CRDs), including very low carbohydrate ketogenic diets (KDs), are increasing in popularity beyond the management of obesity and diabetes. At present, CRDs are being implemented for mental health disorders,^1^, ^2^, ^3^, ^4^ epilepsy, neurodegenerative diseases,^5^^,^^6^ polycystic kidney disease,^7^ and autoimmune and inflammatory conditions,^8^, ^9^, ^10^ to name a few examples. While some of these clinical use cases are backed by human randomized trials, many remain experimental. Nevertheless, there is a clear and rising interest in the therapeutic applications of CRD and KD.

An obstacle to the broad clinical implementation of CRD and KD are lipid changes that occur in a minority of patients upon carbohydrate restriction, characterized by large increases in low-density lipoprotein cholesterol (LDL-C) and associated apolipoprotein B (ApoB). While there are manifold factors contributing to increases in LDL-C and ApoB on CRDs, “leanness” has been shown to be a major source of heterogeneity.^11^^,^^12^ For example, in a recent set of meta-analyses of 41 human randomized controlled trials,^12^ only those with participants with a mean body mass index (BMI) of <25 kg/m^2^ as a group exhibited increases in LDL-C on CRD; those with participants having overweight of class I obesity exhibited no change in LDL-C; and those with participants having class II obesity exhibited decreases in LDL-C. Correspondingly, this meta-analysis also found an inverse association between BMI and LDL-C change; and it also found that having a BMI of <25 kg/m^2^ was >5 times as powerful as being in the top quartile of saturated fat intake for predicting LDL-C change.

These other studies and observations have given rise to the characterization of the lean mass hyper-responder (LMHR),^11^ defined by a triad of elevated LDL-C, along with elevated high-density lipoprotein cholesterol (HDL-C) and low triglycerides that tends to occur in lean, generally healthy individuals adopting a CRD. The phenotype may potentially be explained by the lipid energy model, which is beyond the scope of this report but described in Norwitz et al.^13^

Irrespective of the metabolic and mechanistic drivers of this LMHR phenotype, there is understandable clinical concern, especially among those LMHRs with the most extreme profiles including LDL-C levels in excess of 500 mg/dL with correspondingly high ApoB levels.^14^^,^^15^ However, while clinicians should exercise clinical prudence in their individual practices, the absolute risk associated with the LMHR and near-LMHR phenotypes remains an outstanding question, with no prospective longitudinal data published on this unique population to date (please refer to our prior editorial on conservative clinical management).^16^

In this KETO-CTA study, we followed 100 persons with LMHR or near LMHR phenotypes over 1 year using high-resolution coronary computed tomography angiography (CCTA) with artificial intelligence-guided plaque quantification to characterize plaque progression in this phenotype along with factors that might predict plaque progression. Previously, we had reported that, upon baseline scans, study participants who had been on KD with hypercholesterolemia for a mean of 4.7 years exhibited no greater total plaque score (TPS) compared to a matched control group.^17^

## Methods

### Design and study population

This study was preregistered at Clinical Trials.gov with the code (NCT05733325) and was conducted in compliance with the principles of the Declaration of Helsinki and relevant local laws and regulations. The pre-registered primary outcome was change from baseline NCPV. However, PAV changes are also reported to facilitate comparisons with other cohorts and studies.

Participants were recruited through social media. Interested individuals were then prescreened based on the full eligibility criteria and the availability of supporting medical documentation to confirm serum markers.

The inclusion criteria were

• Being on a KD for ≥24 months
• LDL-C ≤160 mg/dL from the last lipid panel drawn prior to adopting a KD
• LDL-C ≥190 mg/dL on the most recent laboratory on a KD
• An increase of ≥50% in LDL-C after adopting a KD
• HDL-C ≥60 mg/dL
• Triglycerides ≤80 mg/dL
• Glycated hemoglobin <6.0%
• Fasting glucose <110 mg/dL
• High-sensitivity C-reactive protein <2 mg/L

Exclusion criteria were

• Elevated blood pressure (systolic >130 mm Hg, diastolic >80 mm Hg)
• Type 2 diabetes or any lifetime use of antidiabetic medication
• Untreated hypothyroidism (thyroid stimulating hormone >10 mIU/mL)
• Renal insufficiency (calculated creatinine clearance of <50 mL/min with the MDRD [Modification of Diet in Renal Disease Study] equation)
• Liver enzymes >2 times the upper limit of normal at screening visit or total bilirubin >1.5
• Use of medications that elevate LDL-C (anabolic steroids, isotretinoin, immunosuppressant, amiodarone, thiazide diuretics, glucocorticoids, or thiazolidinediones)
• Use of lipid-lowering supplements or medications (statins, red yeast rice, garlic, ezetimibe, berberine, PCSK9 inhibitors)
• Genetically defined familial hypercholesterolemia

### Measurements

All participants were asked to stay on a KD during their follow-up, and to measure adherence, 3 dietary recalls and daily β-hydroxybutyrate (βHB) data were collected using the Automated Self-Administered 24-Hour (ASA24) Dietary Assessment Tool from the National Institutes of Health. Blood βHB monitoring devices by KetoMojo (Napa) were provided to each participant.

All CCTA scans were performed at baseline and 1 year after at The Lundquist Institute for Biomedical Innovation at Harbor-UCLA Medical Center using the 256-multidetector computed tomography (GE Revolution, General Electric) and were blindly read by the level 3 cardiac computed tomography readers. A nonenhanced electrocardiogram-gated coronary artery calcium (CAC) scan was also performed before each CCTA.

Plaque volume quantification was measured using a semiautomated software, Cleerly, and evaluated by experienced readers. This software can detect lumen and vessel border contours automatically, with manual correction by expert readers in any areas of misregistration. Each coronary plaque area identified in at least 2 adjacent slides with a 0.6 mm slice thickness that was assessed by evaluating all affected slides. Plaque volume was then calculated through the multiplication of the area by slice thickness. The summation of the luminal diameter and segments was calculated and is reported as “noncalcified,” “low attenuation,” or “calcified.” This quantitative plaque assessment protocol has been widely used in several studies.^18^ Further methodological details can be found in the published protocol for this study.^19^

LDL-C exposure on a KD was calculated by summing the products of the reported days on a KD prior to study commencement and baseline LDL-C on a KD plus the study follow-up days by their final LDL-C. Estimated lifelong LDL-C additionally included the product of age upon commencing a KD and pre-KD LDL-C. The percent atheroma volume (PAV) was calculated as: (total plaque volume/total vessel volume) × 100.

### Statistical analyses

Data are presented using the median (25th to 75th percentiles) and mean ± SD for continuous variables and count (percentage) for categorical variables. Data cleaning, statistical analyses, and all plots were made using R version 4.0.3 (R Core Team [2020], R Foundation for Statistical Computing, with the last available version for September 2024). Cardiovascular risk was calculated with *CVrisk::chd_10y_mesa*. Linear models on the primary (NCPV) and secondary outcomes were univariable and analyzed using *stats::lm,* and all linear model assumptions were corroborated with the R function *performance::check_model.*

Bayes factors were calculated using *BayesFactor::regressionBF* with default settings and an ∼ *rscale* value of 0.8 to contrast a moderately informative prior with a conservative distribution width (to allow for potential large effect sizes) due to the well-documented association between ApoB changes and coronary plaque changes.^20^

Sensitivity analyses were performed on participants with high diet adherence (defined as 80% βHB measurements ≥0.3) and participants with a 10-year baseline cardiovascular risk >5% assessed with the MESA (Multi-Ethnic Study of Atherosclerosis) equation with ethnicity and CAC inputs (Central Illustration).

**Central Illustration:** **100 Individuals Exhibiting Ketogenic Diet-Induced Low-Density Lipoprotein Cholesterol Elevations Were Followed for 1 Year Using Coronary Artery Calcium and Coronary Computed Tomography Angiography** Neither total exposure nor changes in baseline levels of ApoB and mg/dL were associated with changes in plaque. Conversely, baseline plaque but ApoB was not associated with plaque progression. ApoB = apolipoprotein B; CAC = coronary artery calcium; CCTA = coronary computed tomography angiography; HDL-C = high-density lipoprotein cholesterol; LDL-C = low-density lipoprotein cholesterol; TG = triglycerides.

## Results

All 100 participants completed baseline and follow-up measurements (Supplemental Figure 1). As is characteristic of the LMHR phenotype, mean LDL-C, HDL-C, and triglycerides were 254 ± 85 mg/dL, 89 ± 20 mg/dL, and 67 ± 30 mg/dL, respectively, and mean BMI was 22.5 ± 2.7 kg/m^2^. Mean age was 55.3 ± 10.7 years, and 59% were males (Table 1). While most participants exhibited a TPS of 0 at baseline as assessed by blinded expert inspection (as previously reported^17^), application of modern artificial intelligence-guided CCTA assessment was able to identify quantifiable plaque in all participants at baseline, as expected.

**Table 1:** Baseline Characteristics (N = 100)

Male	59%	
Ethnicity		
Asian	10%	
Hispanic	7%	
White	83%	
Age (y)	55.3 ± 10.6	57.0 (50.8-63.0)
Ketogenic diet duration (d)	1,642.7 ± 913.5	1,427 (1,002-1,938)
Body mass index (kg/m^2^)	22.5 ± 2.7	22.3 (20.6-24.4)
Systolic blood pressure (mm Hg)	121.8 ± 21.1	120 (112-135)
Total cholesterol (mg/dL)	355.1 ± 89.9	338 (301-337)
LDL-C (mg/dL)	253.7 ± 84.7	237 (202-308)
HDL-C (mg/dL)	88.8 ± 20.0	88 (74-102)
Triglycerides (mg/dL)	66.7 ± 30.4	61 (52-77)
Apolipoprotein B (mg/dL)	185.0 ± 50.8	178 (149-214)
Noncalcified plaque volume (mm^3^)	75.9 ± 88.3	44 (15.4-102.3)
Coronary artery calcium score	50.3 ± 100.9	0 (0-54)
Percent atheroma volume	3.2 ± 3.8	1.6 (0.5-4.9)
Total plaque score	1.7 ± 2.6	0 (0-2.0)
10-y CVD risk (MESA_ETH-CAC, %_)	5.2 ± 5.3	3.4 (2.0-5.9)

Values are %, mean ± SD, or median (Q1-Q3). 10-y CVD risk = based on the risk equation from the MESA (Multi-Ethnic Study of Atherosclerosis) with ethnicity and CAC inputs.

CAC = coronary artery calcium; CVD = cardiovascular disease; HDL-C = high-density lipoprotein cholesterol; LDL-C = low-density lipoprotein cholesterol.

Overall participants successfully adhered to their KD as confirmed by detailed dietary assessment (Table 2) and capillary βHB measurements, with 87% of the cohort recording values above ≥0.3 mmol/L on a majority of measurements, a threshold chosen given the known steady-state drop in circulating ketone levels with prolonged adaptation.

**Table 2:** Diet Composition (N = 100)

Carbohydrates (g/d)	39.5 ± 29.8	30.8 (12.6-51.1)
Fat (g/d)	120.2 ± 46.4	113.1 (89.8-139.3)
Saturated fat (g/d)	44.7 ± 18.9	39.4 (29.9-52.6)
Sugar (g/d)	20.2 ± 18.5	11.1 (6.3-22.2)
Fiber (g/d)	6.9 ± 6.5	6.9 (1.3-11.3)
Sodium (mg/d)	3,292.5 ± 1,263.0	2,931.4 (2,217.7-3,265.7)

Values are mean ± SD or median (Q1-Q3). Pooled data from all available dietary records.

No significant changes in either ApoB and BMI were observed after 1 year (median 3 mg/dL, Q1-Q3: −17 to 35 and median −0.2, Q1-Q3: −0.7 to 0.2, respectively.

The median change in NCPV was 18.9 mm^3^ (IQR: 9.3-47.0 mm^3^) and the median change in PAV was 0.8% (IQR: 0.3%-1.7%). Compared to baseline, these represent a 43% and 50% change, respectively. Both NCPV and PAV values were comparable with those observed in other cohorts on both visits (Figures 1A and 1B, Supplemental Table 1).

**Figure 1:** **Individual Change in Plaque Volume** N = 100 individual-level changes in noncalcified plaque volume (NCPV) as measured by artificial intelligence-guided quantification of NCPV at baseline and 1-year follow-up (A). The red line represents the median change (18.9 mm^3^), and the shaded area represents the IQR (9.3-47.0 mm^3^). Compared to baseline, these represent a 43% and 50% change, respectively. (B) The red line represents the median change (0.8%), and the shaded area represents the IQR (0.3%-1.7%).

Neither the change in ApoB throughout the study nor the ApoB level on a KD at the beginning of the study were associated with the change in NCPV (Figures 2A and 2B, Table 3) nor with TPS (Figures 2D and 2E, Table 3).

**Figure 2:** **Changes in Noncalcified Plaque Volume and Total Plaque Score vs Apolipoprotein B and Coronary Artery Calcium** (A to C) Change in ApoB, baseline ApoB, and baseline CAC vs NCPV. (D to F) Change in ApoB, baseline ApoB, and baseline CAC vs NCPV. (G) Final NCPV vs diet LDL-C exposure. (H) ApoB vs saturated fat intake. (C, F) Only CAC is associated with changes in NCPV and TPS. The regression line was fitted with the function “lm,” which regresses y∼x, and the shaded area represents the standard error. ApoB = apolipoprotein B; CAC = coronary artery calcium; LDL-C = low-density lipoprotein cholesterol; NCPV = noncalcified plaque volume; TPS = total plaque score.

**Table 3:** Model Results

	β	*P* Value	R^2^	BF
Estimated LDL-C exposure				
NCPV_final_ ∼ LDL-C_exp_	0.00	0.88	−0.01	(01) 9.9
PAV_final_ ∼ LDL-C_exp_	0.00	0.73	−0.01	(01) 9.1
ApoB				
ΔNCPV ∼ ΔApoB	0.01	0.91	−0.01	(01) >10.0
ΔNCPV ∼ ApoB	0.06	0.33	−0.00	(01) 6.3
Plaque Metrics				
ΔNCPV ∼ CAC_bl_	0.18	<0.001	0.33	(10) >10.0^a^
ΔNCPV ∼ NCPV_bl_	0.25	<0.001	0.49	(10) >10.0^a^
ΔNCPV ∼ PAV_bl_	5.5	<0.001	0.43	(10) >10.0^a^
ΔNCPV ∼ TPS_bl_	7.4	<0.001	0.37	(10) >10.0^a^
ΔNCPV ∼ CAC_bl_∗ ΔApoB				
CAC_bl_	0.18	<0.001	0.33	N/A
ΔApoB	0.08	0.20	N/A	N/A
CAC_bl_: ΔApoB	−0.00	0.23	N/A	N/A
Saturated fat				
ΔNCPV ∼ Saturated fat intake	−0.05	0.77	−0.01	(01) 9.8
ApoB ∼ Saturated fat intake	−0.03	0.90	−0.01	(01) >10.0
Age mediation analysis				
NCPV_final_ ∼ Age	3.0	0.004	0.07	(01) 0.3
NCPV_final_ ∼ Age + Life-LDL-C_exp_	1.93 | 0.01	0.13 | 0.16	0.07	(01) 0.3 | 0.3
NCPV_final_ ∼ Age + Life-LDL-C_exp_ + CAC_bl_	0.02 | 0.01 | 0.73	0.98 | 0.15 | <0.001	0.47	(01) 2.7 | 3.1 | >10.0^a^

β = estimate (slope magnitude); ΔNCPV = change in noncalcified plaque volume; ApoB = apolipoprotein B; ApoB = ApoB on a ketogenic diet; ΔApoB = ApoB change during the study; BF = Bayes factor; CAC_bl_ = CAC at baseline; LDL-C_exp_ = LDL-C exposure while on a ketogenic diet (mean 5.7 y); Life-LDL-C_exp_ = LDL-C exposure over life course to date; NCPV_final_ = noncalcified plaque volume at the end of the study; PAV = percent atheroma volume; R^2^ = squared correlation coefficient (explained variability); TPS_final_ = total plaque score at the end of the study; other abbreviations as in Table 1.

a Models on CAC are provided for the alternative hypothesis (10). All other models are provided for the null hypothesis (01).

By contrast, baseline CAC was positively associated with a change in NCPV (Figure 2C) (β = 1.8, *P* < 0.001, R^2^ = 0.33) (Figure 2F). Similar results were found for other baseline plaque metrics, where baseline NCPV, TPS, and PAV were positively associated with change in NCPV (Table 3).

There was no association between LDL-C exposure while on a KD (mean 5.7 years) and NCPV or TPS (Figure 2G, Table 3). Estimated lifetime LDL-C exposure was only a significant predictor of final NCPV in the univariable analysis but lost significance when age was included as a covariate (Table 3). Both age and lifetime LDL-C exposure lost significance when baseline CAC was included in the model (Table 3).

All associations provided Bayes factors 6 to 10 times more likely under the null (for change in and baseline ApoB vs changes in NCPV) and 10 times more likely under the alternative hypotheses (for baseline plaque metrics [CAC, NCPV, TPS, and PAV] vs changes in NCPV) (Table 3).

Sensitivity analyses on participants with >80% of βHB measurements above 0.3 mmol/L (Supplemental Tables 2 to 4) and with high calculated 10-year cardiovascular risk showed similar results to those just reported (Supplemental Table 5).

## Discussion

While both LDL-C and ApoB are independent risk factors for atherosclerosis, the absolute risk associated with elevated LDL-C and ApoB is context-dependent, including the etiology of the elevations^21^ in these biomarkers as well as interactions with other risk markers.^22^ Thus, these data are consistent with the observation that high LDL-C and ApoB among a metabolically healthy population have different cardiovascular risk implications than high LDL-C among those with metabolic dysfunction, who constitute a majority proportion of the population.^23^

It is worth emphasizing that the population at hand—LMHR and near-LMHR persons on KD—is distinct from any population described previously in several ways.

1) Elevations in LDL-C and ApoB are dynamic and result from a metabolic response to carbohydrate restriction,^13^ rather than as a function of a congenital defect.
2) These participants are of normal healthy weight (BMI <25 kg/m^2^) and metabolically healthy, rather than living with obesity, prediabetes, type 2 diabetes, or other insulin resistance disorders.^11^^,^^14^
3) The high LDL-C and ApoB in this phenotype emerge as part of a lipid triad, also inclusive of high HDL-C and low triglycerides, representing a metabolic signature of a distinct physiological state.
4) The degree of this phenotype appears inversely related to BMI (“leanness”),^12^ consistent with the idea that it is a metabolic response to carbohydrate restriction that is accentuated in leaner, more metabolically healthy persons.

These points are worth emphasizing because unique populations require independent study to properly characterize the risk associated with their metabolic profiles. Furthermore, this is the first and only population in which LDL-C is independently elevated without any clear underlying congenital genetic cause and outside the context of any other notable metabolic dysfunction.

Thus, the LMHR population constitutes a unique and important natural experiment evaluating the lipid heart hypothesis in an unprecedented manner.^16^ The data presented herein are consistent with the notion that elevated ApoB, even at extreme levels, does not drive atherosclerosis in a dose-dependent manner in this population of metabolically healthy individuals with carbohydrate restriction-induced elevations in LDL-C and ApoB.

However, this does not mean that the LMHR population is without risk. While it is true their low-plaque baseline values magnify their percentual changes and the observed absolute NCPV and PAV progression (18.9 mm^3^ and 0.8%, respectively) in this KETO-CTA cohort was comparable to what has been observed in other studies on populations with lower LDL-C across the cardiovascular disease risk spectrum, it should be emphasized that this includes heterogeneity in progression (and regression) across the population.

However, the question that should follow is: “*What explains this heterogeneity?*” Here, ApoB exposure was not a significant predictor of changes in plaque, whereas all baseline plaque metrics were significant predictors of changes in plaque.

At this time, we can only speculate about the lack of association between ApoB and plaque progression and mechanisms driving the progression in this population. Plausible explanations include diet- and health-related differences in lipoprotein quality^24^ and kinetics, insulin sensitivity, or inflammation,^25^ as compared to the general population. Future studies will have to directly assess and compare these potential mechanisms.

These insights can facilitate personalized treatment and risk mitigation strategies based on modern, cost-effective cardiac imaging. For instance, despite profound elevations in LDL-C and ApoB, based on these data, LMHR subjects with CAC = 0 at baseline (n = 57) constitute a low-risk group for PAV progression, even as compared to other cohorts with far lower LDL-C and ApoB. By contrast, LMHR subjects with elevated baseline CAC, possibly from a history of metabolic damage and dysfunction prior to adopting a CRD, appear to constitute a relatively higher risk group for PAV progression even where LDL-C and ApoB are equal to their CAC = 0 counterparts.

The finding that “plaque predicts plaque” could result from underlying susceptibilities in those with greater amounts of pre-existing plaque or could result, more directly, from the proinflammatory state associated with coronary atheroma. More research will be needed to identify the pathophysiology driving the progression of atherosclerosis in people with higher levels of pre-existing plaque.

### Strengths and limitations

A major strength of this study lies in the nature of the participants, who collectively constitute a population of 100 metabolic “outliers,” all characterized by high LDL-C and ApoB in the context of being metabolically healthy and generally lean with drastic changes in LDL-C brought about by carbohydrate restriction. In addition, the dropout rate was 0%, and adherence to the KD was assessed by dietary records and βHB measurements.

Since lack of statistical significance (ie, *P* > 0.05) should not be interpreted as evidence in favor of the null but simply a failure to reject the null, the addition of Bayesian inference adds credence to finding that there is no association between NCPV vs LDL-C or ApoB and TPS vs LDL-C or ApoB. In other words, these data suggest it is 6 to 10 times more likely that the hypothesis of no association between these variables (the null) is true as compared to the alternative.

Of course, this study is not without limitations. The duration of the prospective trial was 1 year. However, given the quality of modern CCTA imaging, it is generally agreed that this is sufficient to observe and quantify changes in NCPV, as we did. Nonetheless, we should mention that the “normal” values for NCPV, PAV, and plaque progression in a healthy population are yet to be fully determined, as there is a wide range of ever-evolving methods, definitions, and analytic techniques. We also do not have a comparator group; however, a carefully matched comparison of 80% of this cohort showed similar and trending lower levels of coronary plaque as compared to other generally healthy populations with lower LDL-C, as reported previously.^17^

## Conclusions

Over a 1-year prospective study of 100 persons exhibiting extreme carbohydrate restriction-induced elevations in LDL-C and ApoB, NCPV increased by 18.9 mm^3^ (IQR: 9.3-47.0 mm^3^). In an exploratory analysis, changes in and baseline levels of ApoB were not associated with changes in NCPV or TPS as measured by CCTA. However, baseline CAC and other plaque metrics were positively associated with increases in coronary plaque, supporting the notion that plaque predicts plaque but ApoB does not.

Perspectives **COMPETENCY IN MEDICAL KNOWLEDGE AND COMMUNICATION SKILLS:** LMHR is an emerging phenotype of growing research interest, with little known previously with respect to mechanism and risk. Physicians’ awareness of unique aspects of the phenotype and unique cardiovascular risk profile can facilitate individualized patient management and future collaborative research effects. Furthermore, patients presenting with the LMHR phenotype often identify with the phenotype and may be more receptive to clinical advice from physicians who acknowledge the unique aspects of their profile, are aware of new and ongoing research in this area, and engage in open discussion of the knowns and unknowns with these patients.

**TRANSLATIONAL OUTLOOK:** Understanding baseline plaque burden in an individual can assist physicians and patients to institute risk mitigation strategies based on modern, cost-effective cardiac imaging. In the opinion of this team, research priorities should include dissecting the driving mechanism behind the LMHR phenotype by testing elements of the lipid energy model, along with comparing lifestyle and pharmacological treat options in LMHR in randomized controlled trials. While these first prospective data should be reassuring for LMHR patients and their physicians, longer-term follow-up (eg, 2-, 5-year CCTA measurements) of this and similar cohorts will also be essential to confirm that LMHR and near-LMHR constitute, as a population, a low cardiovascular risk profile.

## Funding support and author disclosures

This study was funded by the Citizen Science Foundation, 7,320 S Rainbow Blvd, #102 to 182, Las Vegas, NV, United States. Dr Norwitz is coauthor of a Mediterranean low-carbohydrate-diet cookbook; and he donates all royalty payments to nutrition research and education. Dr Feldman has received financial contributions from membership (eg, through Patreon) for continued research and is a partner in Own Your Labs LLC. All other authors have reported that they have no relationships relevant to the contents of this paper to disclose.
